The article "Inhibition of endoplasmic reticulum stress alleviates cigarette smoke-induced airway inflammation and emphysema" was retracted in 2026. Reasons: contaminated cell lines or tissues; concerns about the data.

# Inhibition of endoplasmic reticulum stress alleviates cigarette smoke-induced airway inflammation and emphysema

**DOI:** 10.18632/oncotarget.20768

**Published:** 2017-09-08

**Authors:** Yong Wang, Zhen-Zhen Wu, Wei Wang

**Affiliations:** ^1^ Department of Pneumology, Affiliated Hefei Hospital of Anhui Medical University, Hefei, Anhui, China; ^2^ Department of Immunology, Anqing Medical College, Anqing, Anhui, China; ^3^ Pharmaceuticals, Roche R&D Center (China), Shanghai, China

**Keywords:** cigarette smoke, emphysema, airway inflammation, 4-phenylbutyric acid, apoptosis

## Abstract

Chronic bronchitis and emphysema are pathologic features of chronic obstructive pulmonary disease (COPD). Cigarette smoke (CS)-induced endoplasmic reticulum (ER) stress has been implicated in the COPD development, but the molecular mechanism by which it contributes to COPD etiology and the specific role it plays in COPD pathogenesis remain poorly understood. Here, we aimed to determine the role of ER stress in the pathogenesis of CS-induced airway inflammation and emphysema. Exposure to CS significantly increased the expression of ER stress markers in Beas-2B cells and in mouse lungs, possibly through the production of oxidative stress. Further, inhibition of ER stress by 4-phenylbutyric acid (4-PBA) reduced CS extract-induced inflammation in Beas-2B cells through the modulation of NF-κB signaling. 4-PBA also protected against CS-induced airway inflammation and the development of emphysema in mice, which was associated with a reduction in NF-κB activation and alveolar cell apoptosis in the lungs. Taken together, our results suggest that ER stress is crucial for CS-induced inflammation and emphysema, and that targeting ER stress may represent a novel approach to the treatment of COPD.

## INTRODUCTION

Chronic obstructive pulmonary disease (COPD) is characterized by irreversible airway obstruction, chronic bronchitis, and emphysema [1, 2]. COPD is the major cause of chronic morbidity and mortality worldwide, and will become the third leading cause of death by 2020 [3]. Multiple factors increase the risk for COPD, such as genetic factors and environmental risk factors, of which cigarette smoke (CS) is the most important [4]. Although much is known about COPD, the pathogenesis of COPD is still poorly understood.

The endoplasmic reticulum (ER) is a vast membranous network in the cell that is responsible for protein folding, protein biosynthesis, and post-translational modifications of secretory and membrane proteins [5]. An imbalance in protein folding and protein biosynthesis can lead to the accumulation of unfolded or misfolded proteins in the ER, causing ER stress, which has been implicated in the development of various chronic diseases including obesity, insulin resistance, atherosclerosis, and inflammatory and neurodegenerative diseases [6–10]. The unfolded protein response (UPR) is activated to restore protein homeostasis and is mediated by three ER membrane protein sensors: inositol-requiring protein 1 (IRE1), activating transcription factor-6 (ATF6), and protein kinase RNA-like ER kinase [11]. These sensors regulate ER stress through several signaling cascades and are themselves regulated by the ER chaperone protein, glucose regulated protein 78 (GRP78). Increased ER stress is associated with increased inflammation and apoptotic cell death through the activation of nuclear factor κB (NF-κB) and C/EBP homologous protein (CHOP), respectively.

Recent studies suggest that ER stress plays an important role in the development of COPD [12–15]. However, these studies focus on the detection of ER stress and not on the role of ER stress in the pathogenesis of COPD, which has been largely unexplored. Here, we sought to delineate the molecular mechanisms by which ER stress promotes CS-induced inflammation and emphysema by evaluating the effects of the ER stress inhibitor, 4-phenylbutyric acid (4-PBA), in CS-treated Beas-2B cells and COPD mouse models.

## RESULTS

### CS induces ER stress in human bronchial epithelial cells (Beas-2B) and in mouse lungs

To confirm whether ER stress is activated in response to CS exposure, we examined the expression of GRP78, IRE1α, and CHOP proteins. Western blot analyses showed a time and concentration-dependent induction of IRE1α, GRP78, and CHOP in response to exposure to CS extract (CSE) in Beas-2B cells (Figure 1A and 1B).

**Figure 1:** Cigarette smoke (CS) induces endoplasmic reticulum (ER) stress **(A)** Beas-2B cells were treated with 2% CSE for indicated time. **(B)** Beas-2B cells were treated with indicated concentrations of CSE for 12h. The CSE-induced ER stress was assessed by western blot analyses for IRE1α, GRP78 and CHOP. Western blot analyses represent of 3 independent experiments (A and B). Wild type mice were exposed to air or CS for 3months, and mouse lung homogenate samples were analyzed for the indication of ER stress. **(C and D)** Western blot analyses and densitometric analyses showed enhanced levels of IRE1α, GRP78 and CHOP in CS-exposed mice lungs (lanes 7-12), compared with air exposure (lanes 1-6). Quantification of band intensities were normalized to actin. Bars represent means± SEM. *P < 0.05, **P < 0.01 (Student's t-test). All results represent of 3 independent experiments.

To confirm this ER stress in response to CS in an *in vivo* model, wild type (WT) mice were exposed to air or CS for 3months. After the last treatment, mice were sacrificed and their lungs were extracted. The protein levels of IRE1α, GRP78, and CHOP significantly increased in the lung tissue of mice with chronic CS exposure (Figure 1C and 1D). These results suggest that CS activates ER stress in bronchial epithelial cells and in an animal model of COPD.

### Inhibition of ER stress alleviates CSE-induced inflammation in Beas-2B cells through inhibition of NF-κB signaling

To further evaluate the role of ER stress in CSE-induced inflammation in Beas-2B cells, a chemical chaperone, 4-PBA, was used to inhibit ER stress. Western blot analyses demonstrated that 4-PBA markedly inhibited the CSE-induced increases in IRE1α, GRP78, and CHOP protein expression in Beas-2B cells (Figure 2A). It is well-known that CSE can cause cell death. Cell viability showed that CSE-induced cell death was attenuated by 4-PBA pretreatment (Figure 2B). Interestingly, CSE induced an increase in mRNA and protein expression of IL-6 and IL-8 in Beas-2B cells, which was markedly attenuated in cells pretreated with 4-PBA (Figure 2C and 2D). Moreover, inhibition of ER stress protein by IRE1α siRNA or CHOP siRNA also significantly attenuated the CSE-induced production of IL6 and IL8 (Supplementary Figure 1). Numerous studies have suggested a pivotal role for NF-κB signaling in the regulation of immune and inflammatory responses and it is well established that NF-κB is involved in the CS-induced inflammatory response in the lungs of humans and mice. We next questioned whether 4-PBA could reduce CSE-induced NF-κB activation in Beas-2B cells by examining the expression of p-P65 and the degradation of IκBα, two downstream targets of NF-κB. As shown in Figure 2E, CSE treatment lead to an increase in p-P65 expression and IκBα degradation, both of which were significantly attenuated by pre-treatment with 4-PBA.

**Figure 2:** 4-PBA prevents CSE-induced inflammatory responses in Beas-2B cells through inhibiting NF-κB signaling Beas-2B cells were pretreated with 4-PBA (10mM) or vehicle (PBS) for 12h then stimulated with 2% CSE for 12h **(A, C, D and E)** or indicated concentrations of CSE for 24h **(B)**. (A) Expression of IRE1α, GRP78 and CHOP in Beas-2B cells were detected by Western blot. (B) Cell viability were evaluated by cell counting kit 8 (CCK8) assay. (C) The mRNA expression of IL-6 or IL-8 were analyzed by quantitative PCR. (D) Protein levels of IL-6 or IL-8 in supernatants of cultured Beas-2B cells were analyzed. (E) Expression of phosphorylated-p65 (Nucleus), and IκB in Beas-2B cells were detected by Western blot. Western blot analyses represent of 3 independent experiments. Data are expressed as means ± SEM from 3 independent experiments. *P < 0.05, **P < 0.01 (Student's t-test).

### Oxidative stress mediates CSE-induced ER stress and inflammatory responses

It is well known that CS exposes the lungs to high concentrations of reactive oxidant species, which is an important risk factor for ER stress [16]. We next investigated whether oxidative stress could mediate CSE-induced ER stress and inflammatory responses. Inhibition of oxidative stress by antioxidant NAC efficiently prevented CSE-induced ER stress and reduced the mRNA expression and protein levels of IL6 and IL8 in Beas-2B cells (Figure 3A–3C). Further, NAC inhibited CSE-induced inflammation through the NF-κB pathway (Figure 3D).

**Figure 3:** Role of N-acetylcysteine (NAC) in CSE-induced ER stress and inflammatory responses Beas-2B cells were pretreated with NAC (10mM) or vehicle for 16h then stimulated with 2% CSE for 12h. **(A)** Western blot analyses showed the levels of IRE1α, GRP78 and CHOP. **(B)** Quantitative PCR were performed to analyzed relative mRNA expression of IL-6 or IL-8. **(C)** ELISA measured protein levels of IL-6 or IL-8 in supernatants. **(D)** Expression of phosphorylated-p65 (Nucleus), and IκB in Beas-2B cells were detected by Western blot. Western blot analyses represent of 3 independent experiments. Data are expressed as means ± SEM from 3 independent experiments. *P < 0.05, **P < 0.01 (Student's t-test).

### 4-PBA suppresses CS-induced inflammatory responses in a mouse model of CS exposure

To confirm the relationship between CS and ER stress *in vivo*, we established a mouse model of CS exposure. Mice were administered with PBS or 4-PBA and then exposed to room air or CS for 3 months. Compared to treatment with vehicle, treatment with 4-PBA significantly reduced the levels of ER stress markers in the lung tissues (Figure 4A and 4B). Additionally, 4-PBA treatment prevented CS-induced increase in the protein expression of inflammatory cytokines KC and MIP-2 and in the counts of total leukocytes, macrophages and neutrophils in the bronchoalveloar lavage fluid (BALF) (Figure 4C and 4D). Moreover, western blot analyses showed that CS exposure substantially increased the level of p-P65 in lung tissue and that this increase was prevented by treatment with 4-PBA (Figure 4E).

**Figure 4:** Effect of 4-PBA on CS-induced inflammation in mouse lungs Mice were administered with PBS or 4-PBA and then exposed to room air or CS for 3 months. Representative Western blot analyses of IRE1α, GRP78 and CHOP in mouse lungs, and densitometric analyses of IRE1α, GRP78 and CHOP **(A and B)**. Concentrations of KC, MIP-2 **(C)** and the number of total leukocytes cells, macrophage and neutrophils **(D)** in bronchoalveloar lavage fluid (BALF). Representative Western blot analyses of phosphorylated-p65 in mouse lungs and densitometric analyses of phosphorylated-p65 **(E)**. Quantification of band intensities were normalized to actin. Bars represent means± SEM from 5 mice per group. *P < 0.05, **P < 0.01, ^***^P < 0.001 (Student's t-test).

### 4-PBA protects against CS-induced emphysema and alveolar cell apoptosis

To further assess the role of ER stress in the pathologic processes of COPD, mice were exposed to CS for 6 months and mean linear intercept (Lm) was used to evaluate airspace enlargement. After 6 months of CS exposure, mice displayed significantly augmented airspace in their lungs, which was partly alleviated by 4-PBA treatment (Figure 5A). Similarly, 4-PBA-treated mice resisted CS-induced alveolar cell apoptosis, as revealed by decreased cleaved-caspase 3 staining and TUNEL staining (Figure 5B and 5C). These results suggest that 4-PBA-treated mice are resistant to CS-induced lung inflammation and emphysema.

**Figure 5:** Effect of 4-PBA on CS-induced emphysema and alveolar cells apoptosis in mouse lungs Mice were administered with PBS or 4-PBA and then exposed to room air or CS for 6 months. **(A)** Representative micrographs (n = 10 images per mouse lung; n = 5 mice per group) of mouse lungs with H&E staining and mean linear intercept of mice lungs were measured. Scale bars: 100 μm (insets: 50 μm). **(B)** Representative images (n = 8-10 images per mouse lung; n = 5 mice per group) of immunohistochemistry staining for cleaved caspase-3 in lung section (left). Cleaved caspase-3-positive alveolar septal cells were counted and alveolar cells positive for the Cleaved caspase-3 antibody staining were expressed as a percentage of total cells (right). Scale bars: 50 μm. **(C)** Representative images (n = 8-10 images per mouse lung; n = 5 mice per group) of TUNEL staining in lung section (left). TUNEL-positive alveolar septal cells were counted and alveolar cells positive for the TUNEL staining were expressed as a percentage of total cells (right). Scale bars: 50 μm. Results were shown at means± SEM. *P < 0.05, **P < 0.01, (Student's t-test).

## DISCUSSION

This study demonstrated that CS increased the expression of ER stress markers in airway epithelial cells and mouse lungs. Furthermore, treatment of animals with the ER stress inhibitor 4-PBA significantly alleviated CS-induced airway inflammation, likely via inhibition of NF-κB signaling pathways. 4-PBA also protected against CS-induced airspace enlargement and apoptotic cell death in mouse lungs. Thus, our findings clearly indicate a crucial role for ER stress in the development of CS-induced inflammation and alveolar destruction in COPD, and provide information about a novel mechanism and potential therapeutic target for CS-induced COPD.

Accumulating evidence has suggested that induction of ER stress contributes to the development of pulmonary diseases, including bronchial asthma, lung injury, and idiopathic pulmonary fibrosis [17–19], and that 4-PBA can attenuate ER stress, thus contributing to disease regression. In support of this, administration of 4-PBA has been shown to improve symptom severity in mouse models of bronchial asthma and lipopolysaccharide-induced lung injury [17, 19]. Recent studies also reported an association between ER stress and COPD; exposure to CS induces ER stress in alveolar epithelial cells, mouse lungs, and the lungs of chronic smokers [12–16]. Consistent with previous studies, the current study demonstrated that CS induced the expression of markers of ER stress in airway epithelial cells and mouse lungs. Moreover, pulmonary administration of the ER stress inhibitor 4-PBA inhibited inflammation and emphysema, further illustrating the deleterious role of ER stress in COPD. This study also provided evidence that ER stress in COPD is associated with activation of the NF-κB pathway and induction of lung epithelial cells apoptosis.

Chronic bronchitis is an important feature of COPD, and CS exposure induces airway neutrophilic inflammation in human and mouse models partly through the activation of NF-κB pathways [20, 21]. Neutrophilic inflammation induces the release of proteases and reactive oxygen species, which could ultimately contribute to emphysematous alveolar destruction. Moreover, an increasing body of evidence suggests the presence of a positive feedback loop whereby ER stress immediately activates the inflammatory response, releasing proinflammatory cytokines that in turn induce more ER stress, further amplifying the inflammatory response [22, 23]. In lung injury models induced by LPS [19], viruses [24], or fungus [25], ER stress has been shown to mediate lung inflammation. Consistent with these findings, the current study demonstrated that inhibition of ER stress by 4-PBA effectively alleviated inflammation in cultured Beas-2B cells and in mouse lungs by suppressing NF-κB signaling.

As a key regulator of inflammation, the NF-κB pathway is responsible for the regulation of many proinflammatory cytokines and chemokines involved in different inflammatory processes [26]. Likewise, the NF-κB pathway is involved in the pathogenesis of COPD; expression of NF-κB is associated with the state of COPD [27]. ER stress has been shown to activate NF-κB pathways, partly by translocating NF-κB to the nucleus [28, 29]. Our findings show that ER stress is required for the activation of NF-κB signaling by CS. Taken together, we speculate that the proinflammatory effect of ER stress in CS-induced lung inflammation is mediated by the modulation of NF-κB signaling. However, the precise mechanism by which ER stress activates NF-κB remains poorly understood.

CS contains many reactive oxygen species, carcinogens, and free radicals, all of which are known to trigger ER stress. Kunchithapautham et al. [30] find that pretreatment with NAC can prevent CS-induced activation of GRP78 and CHOP in a human retinal pigment epithelial cell line. Similarly, NAC is also reported to suppress the phosphorylation of ER stress marker eIF2α by CSE in a human lung cancer line [31]. Consistent with previous studies, we showed that NAC inhibited CS-induced ER stress, attenuating the inflammatory response in Beas-2B cells and downregulating the expression of NF-κB. Our study suggests that CS elicits ER stress possibly through the production of oxidative stress and subsequently triggered airway inflammation. Oxidative stress is a pivotal mechanism by which CS mediates the progression of COPD [32, 33]. Antioxidants, such as N-acetylcysteine (NAC), have been shown to prevent exacerbation of COPD [34]. In additional, ER stress and the oxidative stress response have a causal relationship. A recent study showed that 4-PBA can effectively inhibit oxidative stress and that this inhibition may involve ER stress-dependent regulation [35]. It is well established that 4-PBA can improve the folding capacity of ER proteins and facilitate the trafficking of unfolded or misfolded proteins to attenuate ER stress. However, 4-PBA also inhibits ER stress partly through suppressing oxidative stress [35]. Of note, ER stress is just one of cellular and molecular mechanisms for COPD pathogenesis, which explains why 4-PBA failed to completely rescue CS-induced airway inflammation and emphysema ER stress.

Alveolar cell apoptosis is a critical step in the pathogenesis of emphysema [36, 37]. ER stress has been implicated in apoptotic signaling [7] and has been shown to regulate apoptosis in lung epithelial cells and human lung cancer cells [38–40]. Our results are in agreement with these studies in that downregulation of ER stress by 4-PBA decreased CS-induced cell apoptosis, thus preserving alveolar structure. Many studies have verified that CHOP is one of the inducers for apoptosis [41]. However, whether CHOP or other mechanisms regulate alveolar cell apoptosis by CS requires further investigation.

In conclusion, we demonstrated that ER stress is induced and enhances CS-induced airway inflammation and emphysema through the activation of NF-κB and apoptosis. Moreover, pulmonary pathologies induced by CS exposure are markedly attenuated by 4-PBA, suggesting that inhibition of ER stress may serve as a novel therapeutic strategy for COPD.

## MATERIALS AND METHODS

### Cell culture

Human lung Beas-2B cells were purchased from American Type Culture Collection (ATCC) and grown in RPMI 1640 containing 10% fetal bovine serum (FBS) in an atmosphere consisting of 5 % CO2 and 95 % air at 37°C.

### CSE preparation

CSE was prepared by slowly bubbling smoke from Research-grade 1R5F cigarettes (Kentucky Tobacco and Health Research Institute, USA) through 5 ml RPMI 1640, and then filtering it through a 0.22 μm filter. pH was adjusted to 7.4 with NaOH. Then, the sterilized CSE solution was considered as 100% stored at −80 °C.

### Cell viability

Beas-2B cells were plated in the 96-well plates and pretreated with 4-PBA (10mM) or vehicle (PBS) for 12h, then stimulated with different concentrations of CSE(0%, 1%, 2%, 3%) for 24h. Cell viability was evaluated by CCK8 (cell counting kit 8; Dojindo, Tokyo, Japan) assay according to the manufacturer's instructions.

### Reagents

Antibodies to IRE1α, GRP78, CHOP, p-P65, IκB, Cleaved caspase-3 and actin were purchased from Cell Signaling Technology (Danvers, MA). CHOP siRNA, IRE1α siRNA and Control siRNA were purchased from GenePharma (Shanghai, China). Transfection reagent GeneMute were purchased from SignaGen Laboratories. ELISA kits for human IL8, human IL6, mouse KC and mouse MIP-2 were purchased from R&D systems.

### RNA isolation and quantitative real-time PCR (qRT-PCR)

Total RNA from Beas-2B cells was extracted according to the manufacturer's instructions (Qiagen, CA). Total RNA was reverse transcribed using the PrimeScript RT Reagent Kit (Takara, Japan). qRT-PCR was performed with Faststart SYBR Green Kit (Roche, Germany). The relative levels of mRNA were normalized to the expression of actin and analyzed using in relative units.

### Transfection with siRNAs

When cells reached 30%-50% confluence, cells were transfected with 5 nmol siRNA duplexes using transfection reagent GeneMute according to the manufacturer's recommendations.

### ELISA

Cell culture supernatants of IL6 and IL8, and BALF supernatants of KC and MIP-2 collected were used to determine protein levels. ELISA assays were performed using ELISA kits from R&D Systems according to the manufacturer's instructions.

### Western blotting

Beas-2B cells lysates or mouse lung homogenate samples were prepared by lysing them in loading buffer containing RIPA and protease inhibitor cocktail. Then, cells lysates or tissue homogenates were boiled for 8 minutes at 100 °C. After separated by electrophoresis, proteins were transferred onto a polyvinylidene difluoride membranes (PVDF, Millipore), then membranes were blocked with 5% fat-free milk. Afterward, the membranes were incubated with antibodies. Then, the membranes were probed with a secondary antibody and bands were analyzed by a western blot imaging system (Odysey, Li-COR Bioscience).

### Immunohistochemistry staining

Paraffin-embedded inflated lungs were deparafinized and rehydrated. Afterward, endogenous peroxidase in tissue were quenched with 3% H_2_O_2_. The tissue sections were then incubated with antibody according to standard protocols. Images were acquired using an Olympus inverted scope (Olympus, Japan) and staining area were semiquantitatively analyzed with ImageJ software.

### TUNEL

TUNEL was performed using TACS2 TdT DAB kit (Trevigen, USA) according to manufacturer's protocols. Staining area were semiquantitatively analysed with ImageJ software.

### Mice

C57BL/6 mice were purchased from the Animal Center of Slaccas (Shanghai, China). 4-phenylbutyric acid (4-PBA) (20 mg/kg per day, Sigma) diluted with PBS, was intraperitoneal injection twice a week. Mice were exposed to total body CS generated from a smoking chambers for 3 or 6 month, as described [42]. The mice were exposed to 100 cigarettes per day, 2h per day, 5 days per week. At 18h after the last exposure, bronchoalveloar lavage fluid (BALF) was collected and the number of inflammatory cells was counted as described previously [42].

### Lung morphometry

After euthanized, the left lungs were inflated by 4% paraformaldehyde at 25 cm H_2_O pressure and then embedded in paraffin. Lung stained with hematoxylin and eosin (H&E) using standard protocols. The right lungs of mice were removed from the thorax for Western blot analysis. Alveolar size was estimated with the Lm of the airspace as described [43]. In brief, Lm was calculated for each sample based on 10 random fields observed at a magnification of ×200 using a cross-line. Alveoli were considered to be the smallest discrete air spaces bounded by an imaginary straight line. L_T_ is the total test line length. Two kinds of intersections with the test line were counted: 1) visible intersections between alveolar air and adjacent tissue, usually alveolar wall (I_a/w_); 2) visible intersections between alveolar ducts or sacs and adjacent wall (I_d/w_); Lm=2 L_T_/(I_a/w_+ I_d/w_).

### Statistical analysis

Experimental data are expressed as mean ± SEM. GraphPad Prism software (version 4.0; GraphPad software, San Diego) was used to analyze statistical tests. Statistical analyses were performed by the 2-tailed Student t test. P values lower than 0.05 were considered to be statistically significant.

## SUPPLEMENTARY MATERIALS FIGURE



## Abbreviations

4-PBA: 4-phenylbutyric acid
ATF6: Activating transcription factor-6
BALF: Bronchoalveloar lavage fluid
CHOP: C/EBP homologous protein
COPD: Chronic obstructive pulmonary disease
CS: Cigarette smoke
CSE: Cigarette smoke extract
ER: Endoplasmic reticulum
GRP78: Glucose-regulated protein 78
IRE1: Inositol requiring protein 1
NAC: N-acetylcysteine
PKR: Protein kinase RNA
UPR: Unfolded protein response
WT: Wildtype
Lm: mean linear intercept

## References

[1] Barnes PJ, Shapiro SD, Pauwels RA (2003). Chronic obstructive pulmonary disease: molecular and cellularmechanisms. European Respiratory Journal.

[2] Hogg J, Chu F, Utokaparch S, Woods R, Elliott W, Buzatu L, Cherniack R, Rogers R, Sciurba F, Coxson H, Paré P (2004). The nature of small-airway obstruction in chronic obstructive pulmonary disease. N Engl J Med.

[3] Pauwels RA, Rabe KF (2004). Burden and clinical features of chronic obstructive pulmonary disease (COPD). The Lancet.

[4] Barnes PJ (2000). Chronic Obstructive Pulmonary Disease. New England Journal of Medicine.

[5] Gaut J, Hendershot L (1993). The modification and assembly of proteins in the endoplasmic reticulum. Curr Opin Cell Biol.

[6] Hotamisligil GS (2010). Endoplasmic reticulum stress and the inflammatory basis of metabolic disease. Cell.

[7] Appenzeller-Herzog C, Hall MN (2012). Bidirectional crosstalk between endoplasmic reticulum stress and mTOR signaling. Trends in cell biology.

[8] Ozcan L, Tabas I (2016). Calcium signalling and ER stress in insulin resistance and atherosclerosis. Journal of internal medicine.

[9] Pagliassotti MJ, Kim PY, Estrada AL, Stewart CM, Gentile CL (2016). Endoplasmic reticulum stress in obesity and obesity-related disorders: An expanded view. Metabolism: clinical and experimental.

[10] Xiang C, Wang Y, Zhang H, Han F (2017). The role of endoplasmic reticulum stress in neurodegenerative disease. Apoptosis.

[11] Davenport E, Morgan G, Davies F (2008). Untangling the unfolded protein response. Cell Cycle.

[12] Alam S, Li Z, Atkinson C, Jonigk D, Janciauskiene S, Mahadeva R (2014). Z alpha1-antitrypsin confers a proinflammatory phenotype that contributes to chronic obstructive pulmonary disease. American journal of respiratory and critical care medicine.

[13] He B, Luo B, Chen Q, Zhang L (2013). Cigarette smoke extract induces the expression of GRP78 in A549 cells via the p38/MAPK pathway. Molecular medicine reports.

[14] Kenche H, Baty CJ, Vedagiri K, Shapiro SD, Blumental-Perry A (2013). Cigarette smoking affects oxidative protein folding in endoplasmic reticulum by modifying protein disulfide isomerase. FASEB journal.

[15] Geraghty P, Baumlin N, Salathe MA, Foronjy RF, D’Armiento JM (2016). Glutathione Peroxidase-1 Suppresses the Unfolded Protein Response upon Cigarette Smoke Exposure. Mediators of inflammation.

[16] Kelsen SG, Duan X, Ji R, Perez O, Liu C, Merali S (2008). Cigarette smoke induces an unfolded protein response in the human lung: a proteomic approach. American journal of respiratory cell and molecular biology.

[17] Kim SR, Kim DI, Kang MR, Lee KS, Park SY, Jeong JS, Lee YC (2013). Endoplasmic reticulum stress influences bronchial asthma pathogenesis by modulating nuclear factor kappaB activation. The Journal of allergy and clinical immunology.

[18] Korfei M, Ruppert C, Mahavadi P, Henneke I, Markart P, Koch M, Lang G, Fink L, Bohle RM, Seeger W, Weaver TE, Guenther A (2008). Epithelial endoplasmic reticulum stress and apoptosis in sporadic idiopathic pulmonary fibrosis. American journal of respiratory and critical care medicine.

[19] Kim HJ, Jeong JS, Kim SR, Park SY, Chae HJ, Lee YC (2013). Inhibition of endoplasmic reticulum stress alleviates lipopolysaccharide-induced lung inflammation through modulation of NF-kappaB/HIF-1alpha signaling pathway. Scientific reports.

[20] van der Vaart H, Postma DS, Timens W, ten Hacken NH (2004). Acute effects of cigarette smoke on inflammation and oxidative stress: a review. Thorax.

[21] Laucho-Contreras M, Polverino F, Gupta K, Taylor K, Kelly E, Pinto-Plata V, Divo M, Ashfaq N, Petersen H, Stripp B, Pilon A, Tesfaigzi Y, Celli B, Owen C (2015). Protective role for club cell secretory protein-16 (CC16) in the development of COPD. Eur Respir J.

[22] Zhang K, Shen X, Wu J, Sakaki K, Saunders T, Rutkowski DT, Back SH, Kaufman RJ (2006). Endoplasmic reticulum stress activates cleavage of CREBH to induce a systemic inflammatory response. Cell.

[23] Grootjans J, Kaser A, Kaufman RJ, Blumberg RS (2016). The unfolded protein response in immunity and inflammation. Nature reviews Immunology.

[24] Hrincius ER, Liedmann S, Finkelstein D, Vogel P, Gansebom S, Samarasinghe AE, You D, Cormier SA, McCullers JA (2015). Acute Lung Injury Results from Innate Sensing of Viruses by an ER Stress Pathway. Cell reports.

[25] Lee KS, Jeong JS, Kim SR, Cho SH, Kolliputi N, Ko YH, Lee KB, Park SC, Park HJ, Lee YC (2016). Phosphoinositide 3-kinase-delta regulates fungus-induced allergic lung inflammation through endoplasmic reticulum stress. Thorax.

[26] Hayden MS, West AP, Ghosh S (2006). NF-kappaB and the immune response. Oncogene.

[27] Di Stefano A, Caramori G, Oates T, Capelli A, Lusuardi M, Gnemmi I, Ioli F, Chung KF, Donner CF, Barnes PJ, Adcock IM (2002). Increased expression of nuclear factor- B in bronchial biopsies from smokers and patients with COPD. European Respiratory Journal.

[28] Jiang HY, Wek SA, McGrath BC, Scheuner D, Kaufman RJ, Cavener DR, Wek RC (2003). Phosphorylation of the Subunit of Eukaryotic Initiation Factor 2 Is Required for Activation of NF-κB in Response to Diverse Cellular Stresses. Molecular and Cellular Biology.

[29] Deng J, Lu PD, Zhang Y, Scheuner D, Kaufman RJ, Sonenberg N, Harding HP, Ron D (2004). Translational repression mediates activation of nuclear factor kappa B by phosphorylated translation initiation factor 2. Mol Cell Biol.

[30] Kunchithapautham K, Atkinson C, Rohrer B (2014). Smoke exposure causes endoplasmic reticulum stress and lipid accumulation in retinal pigment epithelium through oxidative stress and complement activation. The Journal of biological chemistry.

[31] Jorgensen E, Stinson A, Shan L, Yang J, Gietl D, Albino AP (2008). Cigarette smoke induces endoplasmic reticulum stress and the unfolded protein response in normal and malignant human lung cells. BMC cancer.

[32] Tuder RM, Petrache I, Elias JA, Voelkel NF, Henson PM (2003). Apoptosis and emphysema: the missing link. American journal of respiratory cell and molecular biology.

[33] Pryor W, Stone K (1993). Oxidants in cigarette smoke Radicals, hydrogen peroxide, peroxynitrate, and peroxynitrite. Ann N Y Acad Sci.

[34] Zheng JP, Wen FQ, Bai CX, Wan HY, Kang J, Chen P, Yao WZ, Ma LJ, Li X, Raiteri L, Sardina M, Gao Y, Wang BS, Zhong NS (2014). Twice daily N-acetylcysteine 600 mg for exacerbations of chronic obstructive pulmonary disease (PANTHEON): a randomised, double-blind placebo-controlled trial. The Lancet Respiratory Medicine.

[35] Luo ZF, Feng B, Mu J, Qi W, Zeng W, Guo YH, Pang Q, Ye ZL, Liu L, Yuan FH (2010). Effects of 4-phenylbutyric acid on the process and development of diabetic nephropathy induced in rats by streptozotocin: regulation of endoplasmic reticulum stress-oxidative activation. Toxicology and applied pharmacology.

[36] Petrache I, Natarajan V, Zhen L, Medler T, Richter A, Cho C, Hubbard W, Berdyshev E, Tuder R (2005). Ceramide upregulation causes pulmonary cell apoptosis and emphysema-like disease in mice. Nat Med.

[37] Kasahara Y, Tuder R, Taraseviciene-Stewart L, Le Cras T, Abman S, Hirth P, Waltenberger J, Voelkel N (2000). Inhibition of VEGF receptors causes lung cell apoptosis and emphysema. J Clin Invest.

[38] Nguyen H, Uhal B (2016). The unfolded protein response controls ER stress-induced apoptosis of lung epithelial cells through angiotensin generation. Am J Physiol Lung Cell Mol Physiol.

[39] Liu X, Guo S, Liu X, Su L (2015). Chaetocin induces endoplasmic reticulum stress response and leads to death receptor 5-dependent apoptosis in human non-small cell lung cancer cells. Apoptosis.

[40] Zhang Y, Xu X, Li W, Miao H, Huang S, Zhou Y, Sun Y, Li Z, Guo Q, Zhao L (2016). Activation of endoplasmic reticulum stress and the extrinsic apoptotic pathway in human lung cancer cells by the new synthetic flavonoid, LZ-205. Oncotarget.

[41] Sun SY, Liu X, Zou W, Yue P, Marcus AI, Khuri FR (2007). The farnesyltransferase inhibitor lonafarnib induces CCAAT/enhancer-binding protein homologous protein-dependent expression of death receptor 5, leading to induction of apoptosis in human cancer cells. The Journal of biological chemistry.

[42] Li FF, Shen J, Shen HJ, Zhang X, Cao R, Zhang Y, Qui Q, Lin XX, Xie YC, Zhang LH, Jia YL, Dong XW, Jiang JX (2012). Shp2 plays an important role in acute cigarette smoke-mediated lung inflammation. Journal of immunology.

[43] Kawakami M, Paul J, Thurlbeck W (1984). The effect of age on lung structure in male BALB/cNNia inbred mice. Am J Anat.

